# Effect of Plasma Viremia on Apoptosis and Immunophenotype of Dendritic Cells Subsets in Acute SIVmac239 Infection of Chinese Rhesus Macaques

**DOI:** 10.1371/journal.pone.0029036

**Published:** 2011-12-12

**Authors:** Hou-Jun Xia, Jian-Ping Ma, Gao-Hong Zhang, Jian-Bao Han, Jian-Hua Wang, Yong-Tang Zheng

**Affiliations:** 1 Key Laboratory of Animal Models and Human Disease Mechanisms of Chinese Academy of Sciences and Yunnan Province, Kunming Institute of Zoology, Chinese Academy of Sciences, Kunming, Yunnan, China; 2 Institut Pasteur of Shanghai, Shanghai Institutes for Biological Sciences, Chinese Academy of Sciences, Shanghai, China; 3 Graduate School of the Chinese Academy of Sciences, Beijing, China; George Mason University, United States of America

## Abstract

Non-human primates such as Chinese rhesus macaques (Ch Rhs) provide good animal models for research on human infectious diseases. Similar to humans, there are two principal subsets of dendritic cells (DCs) in the peripheral blood of Ch Rhs: myeloid DCs (mDCs) and plasmacytoid DCs (pDCs). In this study, two-color fluorescence-activated cell sorting (FACS) analyses were used to identify the main DC subsets, namely CD1c^+^ mDCs and pDCs from Ch Rhs. Then, the apoptosis and immunophenotype changes of DCs subsets were first described during the acute phase of SIVmac239 infection. Both the DCs subsets showed decreased CD4 expression and enhanced CCR5 expression; in particular, those of pDCs significantly changed at most time points. Interestingly, the plasma viral loads were negatively correlated with CD4 expression, but were positively correlated with CCR5 expression of pDCs. During this period, both CD1c^+^ mDCs and pDCs were activated by enhancing expressions of co-stimulatory molecules, accompanied with increase in CCR7. Either CD80 or CD86 expressed on CD1c^+^ mDCs and pDCs was positively correlated with the plasma viral loads. Our analysis demonstrates that the pDCs were more prone to apoptosis after infection during the acute phase of SIVmac239 infection, which may be due to their high expressions of CD4 and CCR5. Both DCs subsets activated through elevating the expression of co-stimulatory molecules, which was beneficial in controlling the replication of SIV. However, a mere broad immune activation initiated by activated DCs may lead to tragic AIDS progression.

## Introduction

HIV has been studied for more than 27 years, but it is difficult to understand how the immune systems defend against HIV infection. As a result, an effective vaccine to cure the AIDS could not be developed. A suitable animal model is necessary for HIV study, especially vaccine research and development. Chinese rhesus macaques (Ch Rhs) have been used extensively in recent years to resolve the shortage of Indian-origin rhesus macaques (Ind Rhs), especially in AIDS research. Interestingly, when compared with Ind Rhs, SIVmac pathogenesis in Ch Rhs has been found to be closer to HIV-1 infections in untreated adult humans [1]. Therefore, the Ch Rhs have been considered as a suitable AIDS animal model, and may have advantages over the rapid and highly pathogenic Ind Rhs' model.

Dendritic cells (DCs) are essential for innate and adaptive immunity. In general, DCs patrol around the peripheral tissues of the human body and execute their duty of antigen uptake, process, and presentation to naïve T-cells [2]. DCs are a heterogeneous population, which differ in location, migratory pathways, immunological function, and so on. According to the origin, DCs are divided into two main subsets, namely myeloid DCs (mDCs) and plasmacytoid DCs (pDCs) [3]. mDCs are mostly located in the outside milieu for the detection of pathogens, and form a direct link between innate and adaptive immunity [2], while pDCs are not found in high amounts at sites of pathogen entry. pDCs show a less effective function with regard to capture and presentation than mDCs, and are prone to secrete a large amount of cytokines to influence innate immunity [4].

DCs subsets play a pivotal role in controlling HIV infection and AIDS progression. *In vivo*, numerous studies have shown that the numbers of both mDCs and pDCs are markedly decreased in the blood of patients infected with HIV-1 during the chronic phase [5]–[11], and the DCs are functionally impaired with respect to T-cell proliferation and cytokine production. A decrease in mDCs-associated IL-12 [12] or pDCs-associated IFN-α production [9], [11] was evident in HIV-infected subjects in association with high viral loads and AIDS progression. *In vitro*, the interaction between HIV-1 and DCs is very complicated. On the one hand, both the DCs subsets can be infected by HIV-1 isolates, either R5 or X4 [13]. On the other hand, the DC subsets can be activated by contact with the HIV particles. Human blood pDCs undergo phenotypic and functional activation following exposure to HIV, and induce the bystander maturation of mDCs [14]. The same result that circulating blood DCs subsets increased the surface expression of co-stimulatory molecules was also observed *in vivo* in patients with HIV-1 viremia [6]. However, the activation was influenced by HIV and led to an abnormal immune response. The infected immature MDDCs failed to mature and induced IL-10 production, which caused immune suppression [15].

A large number of evidences demonstrate that chronic, generalized immune activation is a major determinant of AIDS progression in pathogenic HIV-1 and SIVmac infections [16]. The DCs are the initiators of immune activation and are suspected to be the potential factors of AIDS progression. pDCs can sense HIV-1 single-stranded RNA via TLR7 and induce activation of the immune system [17]. It was proved that IFN-α, mainly secreted by HIV-1-stimulated pDCs, has the central role in immune activation and influences disease progression. Meier et al. found that pDCs derived from women produce markedly more IFN-α in response to HIV-1 than those derived from men, which may account for higher immune activation in women. Furthermore, HIV-1-infected women tend to have lower viral loads early, but progress faster to AIDS [18]. Similarly, SIV infection has been found to trigger a rapid and strong IFN-α response in both rhesus macaques and African green monkeys (AGMs) in the acute phase, but only AGMs have been found to effectively control this response and avoid a pathogenic progression [19]. Thus, the activation of pDCs may be predictive of the disease outcome.

Our previous study found that SIVmac239-infected Ch Rhs significantly increased IFN-α and IL-12 production in the acute phase of the infection, which may be the result of an immune activation of DCs subsets [20]. To reveal the *in vivo* status of the DCs subsets, we detected the trend of apoptosis and immunophenotype of CD1c^+^ mDCs and pDCs from Ch Rhs during the acute phase of SIVmac239 infection, and found that pDCs were more influenced by SIV infection than CD1c^+^ mDCs. This discrepancy between pDCs and CD1c^+^ mDCs shows the different roles of DCs subsets in AIDS progression.

## Results

### Phenotypic analysis of Ch Rhs' CD1c^+^ mDCs and pDCs using two-color flow cytometry

The mDCs and pDCs are very rare in blood. In general, human mDCs and pDCs can be identified as Lin^−^HLA-DR^+^CD11c^+^ and Lin^−^HLA^-^DR^+^CD123^+^, respectively. In addition, human DCs also express a group of particular molecules, namely blood dendritic cells antigen (BDCA). The series of BDCA include BDCA-1 (CD1c), -2, -3, and -4. However, only CD1c have been found to show a significant cross-activity with simian PBMCs [21]. CD1c are mainly expressed on the B-lymphocytes and mDCs, and merely a few on monocytes. Therefore, we used CD1c^+^CD14^−^CD20^−^ to estimate the mDCs. Earlier studies have shown that pDCs can be directly recognized as CD123^bright^HLA-DR^+^ cells, either from human [22] or simian [23], [24]. In our study, PBMCs (R1, Figure 1A) were first gated appropriately in the forward-scatter/side-scatter (FSC/SSC) scattergram using FSC as the threshold. The CD1c^+^CD14^−^CD20^−^ of the PBMCs were CD1c^+^ mDCs (R2, Figure 1A), while CD123^bright^HLA-DR^+^ were pDCs (R3, Figure 1A).

**Figure 1:** Two-color strategy for identifying CD1c^+^ mDCs and pDCs. (A) PBMCs (R1) were first gated on Forward-scatter/side-scatter (FSC/SSC) scattergram. Then, CD1c**^+^** mDCs (CD1c**^+^**CD14^−^CD20^−^) were selected in the R2 region and pDCs (CD123^bright^HLA-DR^+^) were selected in the R3 region. (B) The expressions of immunophenotypes, including CD4, CCR5, CD80, CD83, CD86, and CCR7 on DCs subsets were analyzed. Open histograms correspond to isotype controls and filled gray histograms correspond to specific mAbs staining.

Subsequently, the DCs subsets were phenotypically analyzed for other DC and APC markers to ensure the practicable of DCs subdivision through two-color flow cytometry. As shown in Table 1, both CD1c^+^ mDCs and pDCs were negative for linage markers, CD40, CD80, CD83, and DC-SIGN expression, and exhibited low level of CCR7 expression. CD1c^+^ mDCs expressed a high percentage of CD86, while pDCs expressed low. pDCs lacked most of the myeloid markers, such as CD11b and CD11c. In humans, the CD11c^+^ mDCs can be subdivided into three different subsets, namely, CD16^+^, CD1c^+^, and BDCA-3^+^ mDCs [25]. However, the CD1c^+^ mDCs of Ch Rhs have been found to show almost no expression of CD11c. Brown et al. pointed that the CD11c^+^ mDCs of Ind Rhs exhibit no expression of CD1c [26], similar to our results. It is very different from the SIV-receptors expressions of CD1c^+^ mDCs and pDCs; the pDCs highly expressed CD4 and CCR5, which were quite low on CD1c^+^ mDCs. A representative experiment for the expression of SIV receptors and activation markers on DCs subsets is depicted in Figure 1B.

**Table 1:** Phenotypic analysis of CD1c^+^ mDCs and pDCs subsets identified by two-color flow cytometry.

Marker	CD1c^+^ mDC	pDC
Lineage		
CD3	**−**	**−**
CD8	**−**	**−**
CD14	**−**	**−**
CD16	**−**	**−**
CD20	**−**	**−**
APCs		
CD40	**−**	**−**
CD80	**−**	**−**
CD83	**−**	**−**
CD86	**+**	**−/+**
HLA-DR	**+**	**+**
Integrins		
CD11b	**−/+**	**−**
CD11c	**−/+**	**−**
HIV receptor		
CD4	**−/+**	**+**
CCR5	**−/+**	**+**
DC-SIGN	**−**	**−**
Migration		
CCR7	**−/+**	**−/+**

−: negative expression (less than 1% positive cells).

−/+: marginal positive expression (less than 30% positive cells).

+: positive expression (more than 90% positive cells).

### The percentage of pDCs, not CD1c^+^ mDCs, showed transient increase during acute SIVmac239 infection

Four Ch Rhs were infected with SIVmac239, and the viral loads (Figure 2A) have been described in a previous study [20].

**Figure 2:** The dynamics of viral loads and DC subsets percentages in Ch Rhs during primary SIVmac239 infection. (A) Plasma viral loads in SIVmac239-infected Ch Rhs; (B) Blood CD1c**^+^** mDCs percentages in PBMCs during the infection; (C) Blood pDCs percentages in PBMCs during the infection.

The percentage of CD1c^+^ mDCs in PBMCs before infection was 0.62±0.05%, which declined to a nadir (0.36±0.14%) at the day 15 p.i. Then, the value returned and fell again. Furthermore, CD1c^+^ mDCs did not show a significant increase or decrease during this period (Figure 2B). However, the percentage of pDCs in PBMCs was significantly increased at days 6 (0.23±0.08%, *P* = 0.05) and 34 (0.26±0.08%, *P* = 0.046), compared with the normal value (0.12±0.05%) before infection. These increases may be due to the migration of the pDCs into the blood and the loss of CD4^+^ T-cells (Figure 2C).

### Increased apoptosis of pDCs, not CD1c^+^ mDCs, during acute SIVmac239 infection

In our previous study, we found that the absolute numbers of both the DCs subsets decreased to a nadir at day 15 p.i [20]. A potential mechanism for this phenomenon could be a high rate of cell death. Therefore, simian PBMCs stained with Annexin V were used to identify the DCs subsets undergoing apoptosis. Before infection, the percentage of Annexin V positive CD1c^+^ mDCs (31.7±4.0%) was obviously higher than apoptotic pDCs (1.4±0.5%). However, the apoptosis of CD1c^+^ mDCs was not significantly alter during the acute phase of infection, despite the fact that there was a little increase on most of the days, when compared with the day before infection (Figure 3A). Apoptosis of pDCs was significantly influenced by SIVmac239 infection. When compared with pre-infection, the percentage of Annexin V positive pDCs significantly increased at days 15 (6.0±1.8%, *P* = 0.05) and 34 p.i (16.0±1.0%, *P* = 0.001) (Figure 3B). This demonstrates that the virus selectively induced apoptosis of pDCs, rather than CD1c^+^ mDCs.

**Figure 3:** The dynamics of CD1c^+^ mDCs and pDCs apoptosis in Ch Rhs during primary SIVmac239 infection. (A) The percentages of apoptotic CD1c**^+^** mDCs in PBMCs during infection; (B) The percentages of apoptotic pDCs in PBMCs during infection.

### Effect of SIVmac239 on blood CD1c^+^ mDCs and pDCs expression of CD4 and CCR5 during acute infection

Most of the studies have shown that the isolated blood DCs subsets expressed CD4 and CCR5, and can be directly infected by HIV [13], [27]. Simian DCs subsets also expressed these SIV receptors [28], [29]. As shown in Figure 1B, CD1c^+^ mDCs from Ch Rhs had a low expression of CD4 and CCR5. However, almost all pDCs expressed CD4 and CCR5, which seem to imply that the pDCs were more susceptible to SIVmac239 infection than CD1c^+^ mDCs. Subsequently, the mean fluorescence intensities (MFI) of CD4 and CCR5 expressed on both CD1c^+^ mDCs and pDCs were observed during the acute SIVmac239 infection (Figure 4A). Because of the low percentage of CD4 and CCR5 expression, the CD1c^+^ mDCs showed a low MFI of both CD4 and CCR5 which represented a background staining. The MFI of CD1c^+^ mDCs' CD4 was not obviously changed. The expression of CCR5 on CD1c^+^ mDCs increased at day 10, but was not significant. On the other hand, pDCs those highly expressed CD4 and CCR5 were prone to be influenced by SIV infection. At the baseline, the value of pDCs' CD4 MFI was 21.18±1.93, which was significantly decreased at days 3 (16.77±2.83, *P* = 0.039), 6 (16.05±3.29, *P* = 0.049), 15 (11.37±1.59, *P* = 0.05), 19 (12.06±2.18, *P* = 0.002), 27 (14.55±1.89, *P* = 0.001), 34 (15.58±0.96, *P* = 0.01), and 62 (12.34±3.05, *P* = 0.028) p.i. This indicates that the SIVmac239 infection downregulated the expression of CD4 on pDCs. On the contrary, the CCR5 MFI of pDCs was significantly increased at days 6 (84.05±13.13, *P* = 0.018), 10 (127.29±17.39, *P* = 0.01), 15 (115.77±14.54, *P* = 0.005), 19 (155.48±21.87, *P* = 0.005), 27 (169.10±28.59, *P* = 0.013), 34 (92.20±9.15, *P* = 0.001), and 62 (85.95±15.01, *P* = 0.039) p.i from the basic value (47.33±8.26). This was propitious to mobilizing the migration of pDCs to the infected sites and increasing the probability of infection by SIV.

**Figure 4:** Dynamics of SIV receptor expression on CD1c^+^ mDCs and pDCs during primary SIVmac239 infection and their associations with plasma viral loads. (A) Sequential changes of the MFI of CD1c^+^ mDCs CD4, CD1c^+^ mDCs CCR5, pDCs CD4, and pDCs CCR5 after SIVmac239 infection. (B) Analysis of correlations between plasma viral loads and the MFI of CD1c^+^ mDCs CD4, CD1c^+^ mDCs CCR5, pDCs CD4, and pDCs CCR5. NS: not significant.

Subsequently, the correlations between the dynamics of CD4 or CCR5 expression on both the DCs subsets and virus loads were analyzed (Figure 4B). There were no statistical correlations between CD4 and CCR5 expression on CD1c^+^ mDCs and virus loads during infection. However, the CD4 expression on pDCs was negatively correlated with the viral loads (*r* = −0.365, *P* = 0.02), while the CCR5 expression on pDCs was positively correlated with the viral loads (*r* = 0.461, *P* = 0.003).

### Effect of SIVmac239 on blood CD1c^+^ mDCs and pDCs expression of co-stimulatory molecules during acute infection

When activated, the DCs upregulated the expression of co-stimulatory molecules, such as CD80 and CD86 [2]. *In vitro*, the HIV particles, irrespective of whether active or inactive, stimulated the DCs subsets to upregulate the expressions of co-stimulatory molecules [30], [31]. In normal Ch Rhs, the CD1c^+^ mDCs expressed low CD80 and moderate CD86, and pDCs expressed low CD80 and CD86 (Figure 1B). Furthermore, both the DCs subsets presented an immature status.

During the acute SIVmac239 infection, the percentage of CD80^+^ CD1c^+^ mDCs increased from 1.36±0.24% to the peak at day 10 (15.25±8.61%) and sustained a high percentage till day 19 (3.93±0.48%), and showed a significant increase at day 19 (*P* = 0.011). The CD86^+^ CD1c^+^ mDCs maintained a high percentage all the time and showed no obvious change (Figure 5A). The percentage of CD80^+^ pDCs also increased to a peak at day 15 (16.09±3.70%) and showed a significant increase at day 48 (13.44±2.35%, *P* = 0.021), when compared with that before infection (4.07±1.19%). Similarly, the percentage of CD86^+^ pDCs presented an ascending trend and achieved a peak at day 15 (23.11±4.53%) p.i (Figure 5A). Through the analysis of correlation, both CD80^+^ pDCs (*r* = 0.462, *P* = 0.003) and CD86^+^ pDCs (*r* = 0.359, *P* = 0.023) were found to show a positive correlation with the time of infection, which seems to imply that more and more pDCs are activated following disease progression. This phenomenon was not found in CD1c^+^ mDCs. However, both the percentage of CD80^+^ pDCs and CD86^+^ pDCs decreased at day 6, which may be related to the rapid influx of fresh pDCs into the blood, as described in previous studies [20], [32].

**Figure 5:** Dynamics of co-stimulatory molecules expression on CD1c^+^ mDCs and pDCs during primary SIVmac239 infection and their associations with plasma viral loads. (A) Sequential changes of the percentage of CD1c^+^ mDCs CD80, CD1c^+^ mDCs CD86, pDCs CD80, and pDCs CD86 after SIVmac239 infection. (B) Analysis of correlations between plasma viral loads and the percentage of CD1c^+^ mDCs CD80, CD1c^+^ mDCs CD86, pDCs CD80, and pDCs CD86. NS: not significant.

Further, the analysis of correlations between the expression of co-stimulatory molecules on DCs subsets and virus loads was carried out (Figure 5B). While the percentage of CD86^+^ CD1c^+^ mDCs was not correlated with the viral loads, the percentage of CD80^+^ CD1c^+^ mDC (*r* = 0.469, *P* = 0.002), CD80^+^ pDC (*r* = 0.409, *P*  = 0.009), and CD86^+^ pDC (*r* = 0.422, *P*  = 0.007) were positively correlated with the viral loads. Noticeably, the expression of CD86 on CD1c^+^ mDCs was not only high, but also showed increased value of MFI (Figure 6A). Interestingly, the MFI of CD86 on CD1c^+^ mDCs also showed a positive correlation with the virus loads (*r* = 0.352, *P* = 0.026) (Figure 6B).

**Figure 6:** The effects of SIV on the MFI of CD1c^+^ mDC CD86 after SIVmac239 infection. (A) The dynamics of CD86 MFI on CD1c**^+^** mDCs; (B) Analysis of correlation between plasma viral loads and the MFI of CD1c**^+^** mDCs CD86.

### Effect of SIVmac239 on blood CD1c^+^ mDCs and pDCs migration during acute infection

Once activated by virus, the DCs were found to undergo progressive maturation and migration, and the migrated DCs elevated the expression of CCR7. Most of the freshly isolated DCs expressed less than 10% of CCR7 (Figure 1B). As shown in Figure 7A, the percentage of CCR7^+^ CD1c^+^ mDCs obviously increased and showed a significant increase at days 48 (12.74±3.56%, *P = *0.021) and 62 (6.53±1.60%, *P = *0.043) p.i, when compared with that during pre-infection (2.40±1.71%), while the percentage of CCR7^+^ CD1c^+^ mDCs was negatively correlated with that of CD1c^+^ mDCs in PBMCs (*r* = −0.375, *P*  = 0.017). The percentage of CCR7^+^ pDCs obviously increased at day 6, but it was not significant, because just two of the four Ch Rhs showed elevated expression of CCR7 (#04029: 71.82%; #05049: 45.83%; Figure 7B). In addition, neither the percentage of CCR7^+^ CD1c^+^ mDCs nor CCR7^+^ pDCs was correlated with the virus loads.

**Figure 7:** Dynamics of CCR7 expression on CD1c^+^ mDC and pDC during primary SIVmac239 infection. (A) The dynamics of CCR7 expression on CD1c^+^ mDC; (B) The dynamics of CCR7 expression on pDC.

## Discussion

SIV-infected non-human primates can simulate the pathogenesis of HIV infection, and were popularly used all over the world. Now, non-human primates/AIDS models can be divided into two groups, namely, the nonpathogenic SIV infection in natural hosts (Sooty mangabey and AGMs) and the pathogenic SIV infection in rhesus macaques and cynomolgus macaques. A large and growing body of evidence suggests that a chronic, generalized immune activation is a major determinant of disease progression in pathogenic SIVmac infection, similar to humans [33]. The natural hosts routinely maintain a low level of immune activation, which prevents chronic immune exhaustion and progression to AIDS [34].

The DCs play a pivotal role in initiating the immune activation. In this study, we analyzed the effect of plasma viremia on apoptosis and immunophenotype of DCs subsets in acute SIVmac239 infection of Ch Rhs. Through two-color flow cytometry, we gated the mDCs using CD1c^+^CD14^−^CD20^−^. As a myeloid marker, CD1c belongs to the CD1 family, which mediates lipid presentation. Later, studies have pointed out that a specific blood mDC marker, namely BDCA-1, is CD1c. Besides BDCA-1, there are three other BDCA proteins expressed on the DCs subsets. However, only the antibody of BDCA-1 can cross-react with rhesus macaques [21]. The CD1c are mainly expressed on mDCs and B-lymphocytes. However, a little amount of the simian CD1c are expressed on the monocytes, and hence, we added the CD14 antibody to eliminate its influence. Piccioli et al. [25] divided the Lin^−^HLA^−^DR^+^CD11c^+^ mDCs from humans into CD1c, CD16, and BDCA-3 mDCs; however, the same mDCs from Ind Rhs do not express CD1c [26]. Our results also showed that the CD1c^+^ mDCs from Ch Rhs expressed low level of CD11c, indicating that the CD1c^+^ mDCs are different from the traditional CD11c^+^ mDCs in Ch Rhs. CD123^bright^HLA-DR^+^ can be directly used to identify the pDCs, described in human [22] and simian [23], [24] researches. Furthermore, immunophenotype detection has demonstrated that both the DCs subsets showed no expressions of lineage markers. Therefore, the two-color method can be used to identify the DCs subsets. The expressions of CD4 on human mDCs and pDCs were found to be high, while that of CCR5 presented a controversial conclusion in different studies [8], [13], [35]. In Ch Rhs, CD1c^+^ mDCs expressed low level of CD4 and CCR5, which were different from human and simian CD11c^+^ DCs, and hence, they may be a new subset of mDCs. The expressions of CD4 and CCR5 on pDCs of Ch Rhs were similar to those of Ind Rhs [28]. According to the SIV receptors, it is obvious that pDCs are more susceptible to SIV infection than CD1c^+^ mDCs. It has been confirmed that an increased percentage of Annexin V^+^ pDCs is significant during acute SIVmac239 infection, when compared with that of pre-infection, while no significant change could be found in CD1c^+^ mDCs.

After infection, the MFI of CD4 on DCs subsets showed a tendency to decrease, while that of CCR5 showed a contrary tendency to increase. At most of the days, the CD4 and CCR5 expressed on pDCs showed significant changes, when compared with that during pre-infection. It is already known that CD4 is the receptor of HIV/SIV. After the establishment of productive infection, the presence of CD4 has been found to disrupt the life cycle of the virus, including the possibility of super-infection, premature binding of CD4 to nascent virus particles, and inhibition of virus release [36]. However, virus has overcome these problems by downregulating CD4 expression and/or degrading the newly synthesized CD4 protein. An earlier paper has pointed out that Nef of HIV mediated the internalization of the surface CD4 into the endosomes and transferred them to lysosomes for degradation after HIV infection [37]. *In vivo,* Barron et al. [6] found that both the absolute number and percentage of CD4^+^ DCs in Lin^-^HLA-DR^+^ cells were significantly decreased in HIV-infected patients, and the percentage of CD4^+^ DCs was negatively correlated with the plasma HIV RNA; however, this was not significant when detecting the mDCs and pDCs, respectively. In our study, the MFI of CD4 on pDCs was negatively correlated with the virus loads, which indicated that the increase in the virus load leads to more and more infected pDCs downregulating the CD4 expression. However, this correlation was not found in CD1c^+^ mDCs CD4 expression.

The CCR5 expression increased along with the disease progression. *In vitro*, HIV Nef mediated CCR5 endocytosis and degradation [38]. In addition, the DCs downregulated the CCR5 expression and upregulated the CCR7 expression after being stimulated by HIV [39]. *In vivo*, Barron et al. [6] pointed out that the MFI of mDCs CCR5 was higher in HIV-infected patients, while that of pDCs showed no difference. However, in another study, Almeida et al. [5] found that both the percentage and MFI of CCR5 expressed on pDCs were significantly lower in HIV progressors. During the acute phase of infection, the MFI of pDCs CCR5 significantly increased at most of the infectious time points, which was different from the results observed on humans. This may be due to the different period of samples collection. Noticeably, the increase in the CCR5 intensity was observed to be accompanied by an increased probability of infection. It has been reported that the intensity of CCR5 expressed on CD4^+^ T-cells determines the virus load in HIV-1-infected persons, and that there is a strong positive correlation between HIV RNA plasma level and CCR5 density without cell activation and HIV-induced CCR5 upregulation [40]. This phenomenon was also observed in SIVmac239-infected Ch Rhs, where the MFI of pDCs CCR5 was positively correlated with the virus loads. However, the intensity of CD4^+^ T-cells CCR5 was not decreased after highly active antiretroviral therapy (HAART) [40], which indicates that the elevation of CCR5 leads to increase in the virus load, and not vice versa. It has been found that CCR5 is not only the co-receptor of HIV/SIV, but also the ligand of chemokine CCL5 that may promote the DCs migrating to the inflammatory sites after stimulation [4]. HIV-Infected pDCs can secrete high level of RANTES/CCL5 [35], and hence, there an increased concentration of CCL5 secreted by SIV-infected pDCs might induce other normal pDCs to upregulate CCR5 and migrate to the infectious sites, leading to more and more infected pDCs.

Subsequently, we detected the influence of plasma virus loads on DCs' activation and migration. The normal blood DCs maintained an immature status and expressed low co-stimulatory molecules. *In vitro*, HIV infection can induce pDCs to upregulate the expression of CD80, CD86, and CCR7, and promote the bystander maturation of mDCs by secreting a large amount of IFN-α [14]. Similarly, increased surface expression of co-stimulatory molecules was observed on both the DCs subsets in HIV-1 infected patients. Barron et al. pointed out that Lin^−^HLA^−^DR^+^ DCs expressed more CD86 and CD40 in HIV-1-infected viremic subjects, and the MFI of CD86 was positively correlated with the plasma HIV RNA levels, while negatively correlated with CD4^+^ T-cells counts [6]. Subsequently, Dillon et al. [41] showed a partial activation of circulating DCs from viremic HIV-1-infected donors. Although the expression levels of CD40, CD83, and CD86 on DCs subsets increased, only the mDCs CD40 expression presented a significant change. The CD40 expression on both mDCs and pDCs was positively correlated with the virus loads. In our study, the expression of CD80 and CD86 on both CD1c^+^ mDCs and pDCs also increased between days 10 and 15 p.i. Except CD86^+^ CD1c^+^ mDCs, the percentage of CD80^+^ CD1c^+^ mDCs, CD80^+^ pDCs, and CD86^+^ pDCs was positively correlated with the virus loads. Further analysis showed that the MFI of CD86^+^ CD1c^+^ mDCs was also positively correlated with the virus loads. These results indicate that the DCs subsets are activated during the acute phase of infection and migrate to the lymph nodes for initial immune response. However, the DCs in the lymph nodes were found to undergo incomplete maturation and exhibit reduced expression of CD80 and CD86 [42], [43]. In Ind Rhs with AIDS, this activation of blood DCs subsets was not observed, indicating impaired activation of DCs in the late phase [44]. The CCR7 expression accompanied by the activation was significant on the CD1c^+^ mDCs. The CCR7 on pDCs increased to a peak at day 6 p.i, which is earlier than that in Ind Rhs [45].

In summary, our study focused on the influence of SIVmac239 on the status of DCs subsets from Ch Rhs during the acute phase of infection. The results revealed that the pDCs were more prone to apoptosis after infection, which may be due to their high expressions of CD4 and CCR5. Both the DCs subsets showed decreased CD4 expression and enhanced CCR5 expression; particularly, those of pDCs significantly changed at most of the time points. The MFI of CD4 expressed on pDCs was negatively correlated with the plasma viral loads, while the MFI of CCR5 was positively correlated. However, no correlation was found in CD1c^+^ mDCs. During this period, the percentage of active CD1c^+^ mDCs and pDCs obviously increased, following an increase in CCR7. Either CD80 or CD86 expressed on CD1c^+^ mDCs and pDCs was positively correlated with the plasma viral loads. The activation of DCs was found to be beneficial in controlling the replication of SIV. However, a mere broad immune activation initiated by activated DCs may lead to tragic AIDS progression.

## Materials and Methods

### Animals

#### Ethics Statement

All animal and in vitro procedures were performed using standard protocols and according to guidelines approved (Approval number: 20070430) by the Ethics Committee of Kunming Institute of Zoology, Chinese Academy of Sciences in accordance with the recommendations of the Weatherall report. "The use of non-human primates in research".

Four adult male Ch Rhs (*Macaca mulatta*) were obtained from the Kunming Primate Research Center, Chinese Academy of Sciences (CAS). Naïve animals were screened and found to be negative for simian type D retrovirus (SRV) and SIV using antibody ELISA and PCR prior to use. All the four Ch Rhs (05049, 04029, 04039, and 01035) were inoculated intravenously with 5×10^3^ 50% tissue culture infectious doses of SIVmac239, and observed only during the early phase of infection, probably 62 days p.i.

### Viral loads

The levels of viral RNA in plasma were measured by an in-house real-time PCR method as previously described [20].

### Flow cytometric analysis

Two-color fluorescence-activated cell sorting (FACS) analysis was used to identity the DCs subsets. Unlike the common method, CD1c^+^CD14^−^CD20^−^ were used to gate the CD1c^+^ mDCs, and CD123^bright^HLA-DR^+^ were used to gate the pDCs. Subsequently, the immunophenotype of mDCs and pDCs from whole blood samples of naïve and SIV-infected monkeys was detected by three-color flow cytometry using the residual fluorescent channel. In brief, the whole blood (100 µl) was incubated with the appropriate monoclonal antibodies against CD1c (clone AD5-8E7; Miltenyi), CD3ε (clone SP34; BD), CD4 (clone MT-466; Miltenyi), CD8 (clone BW/135/80; Miltenyi), CD11b (clone M1/70.15.11.5; Miltenyi), CD11c (clone 3.9; eBioscience), CD14 (clone M5E2; Biolegend), CD14 (clone TÜK4; Miltenyi), CD16 (clone VEP13; Miltenyi), CD20 (clone 2H7; Biolegend), CD20 (clone LT20; Miltenyi), CD40 (clone 5C3; BD), CD80 (clone L307.4; BD), CD83 (clone HB15e; BD), CD86 (clone FUN-1; BD), CD123 (clone 7G3; BD), CD209 (clone 120507; R&D), CCR5 (clone 3A9; BD), CCR7 (clone 150503; R&D), HLA-DR (clone G46-6; BD), and HLA-DR (clone L243; BD) for 15 min at room temperature. Then, 1 ml of FACS lysing solution (BD Biosciences) was added to each sample to lyse the red blood cells and fix the samples. The remaining cells were washed at 500×g for 5 min. The cell pellet was re-suspended in Dulbecco's PBS with BSA (DPBS-BSA BD) for flow cytometric analysis. Appropriate isotype-matched control antibodies were used in all the labeling experiments. Almost 300,000 events of each sample were acquired through the FACS Calibur flow cytometer (Becton Dickinson) and analyzed using CellQuest software.

### Apoptosis detection of DCs subsets

Simian peripheral blood mononuclear cells (PBMCs) were isolated from monkeys by Ficoll-Paque (GE Healthcare) density gradient centrifugation and adjusted to 1×10^7^ cells/ml. And 1×10^6^ cells were precipitated and re-suspended in 100 µl of DPBS-BSA. A mixture of antibodies used to identify mDCs (CD1c/CD14/CD20) and pDCs (CD123/HLA-DR) were added. After incubating in the dark for 30 min at 4°C, simian PBMCs were washed and stained with Annexin V (Bender MedSystems) in binding buffer for another 10 min. The apoptosis of DCs subsets were detected and analyzed using an FACS Calibur flow cytometer.

### Statistical analysis

All data were analyzed using SPSS 13.0 software. Baseline and follow-up data were compared using the paired t-test or Wilcoxon matched-pairs test, according to the distribution of the variables analyzed by Shapiro-Wilk test. The nonparametric Spearman's rank correlation test was used to investigate the relationship between the parameters. For all the tests, two-sided p<0.05 was considered to be significant.
